# Exploring the Mechanism of Realgar against Esophageal Cancer Based on Ferroptosis Induced by ROS-ASK1-p38 MAPK Signaling Pathway

**DOI:** 10.1155/2022/3698772

**Published:** 2022-09-12

**Authors:** Ruyi Yang, Fazhang Chen, Haizhen Xu, Zhanfang Guo, Changxia Cao, Hongyan Zhang, Changrong Zhang

**Affiliations:** ^1^Department of Integrative Medicine, Affiliated Hospital of Qinghai University, Xining 810001, Qinghai, China; ^2^Medical College of Qinghai University, Xining, China

## Abstract

**Background:**

Realgar (REA), a Chinese herbal decoction, has been used to treat various tumors and has produced positive outcomes; however, there is a lack of convincing evidence for the treatment of esophageal cancer. The present study aimed to investigate the effects of REA on esophageal cancer (EC) and explore its mechanism.

**Methods:**

EC cells Eca109 and KYSE150 were selected for this study, and different groups of treated cells were set up. We studied the inhibition rate and half inhibition concentration (IC_50_) by CCK-8 method, the clone formation assay was used to detect the clone formation ability, the scratch assay is used to determine the cell migration ability, the Transwell assay was used to detect the cell invasion ability, the protein expressions of E-cadherin, Slug, N-cadherin, ASK1, p38 MAPK, p-p38 MAPK, and GPX4 were determined using Western blot, the mRNA expressions of ASK1 and p38 MAPK were assessed using qRT-PCR, transmission electron microscopy was used to observe the cellular ultrastructure, Prussian blue staining was used to observe the intracellular iron particle distribution, and biochemical analysis of cellular MDA, SOD, GSH, and GPXS activities, flow cytometric analysis of cellular ROS levels, immunofluorescence staining to detect cellular GPX4 expression, and JC-1 method to detect mitochondrial membrane potential were used.

**Results:**

REA inhibited the proliferation of Eca109 and KYSE150 cells in a time- and concentration-dependent manner, and REA significantly inhibited the migration and invasion of Eca109 and KYSE150 cells and activated the cellular ferroptosis and ROS-ASK1-p38 MAPK signaling pathways (*P* < 0.05). Inhibition of activation of the ROS-ASK1-p38 MAPK signaling pathway promoted the inhibition of proliferation, migration, and invasion of Eca109 and KYSE150 cells and the induction of ferroptosis by REA.

**Conclusion:**

REA induced ferroptosis and inhibited the migration of EC cells by activating the ROS-ASK1-p38 MAPK signaling pathway.

## 1. Introduction

Esophageal cancer (EC) is the third most prevalent cancer and the fourth most deadly cancer in China [1]. EC is not easy to be diagnosed early and has a poor prognosis and a low 5-year survival rate after surgery [2]. Chemotherapy combined with radiotherapy is the most common clinical treatment for EC. However, these treatments are prone to drug resistance and a series of toxic side effects, such as kidney damage, bone marrow suppression, leukocyte decline, and thrombocytopenia [3]. Therefore, there is an urgent need to develop anti-EC drugs with good efficacy and low toxic side effects.

Currently, herbal medicines are attracting attention as a new source of anticancer drugs [4]. Among them, Xionghuang (Realgar, REA) is an herbal medicine containing arsenic compounds, which has been widely used in Chinese medicine for many years [5]. Studies have shown that REA has analgesic, anti-inflammatory, immune-enhancing, and other effects, and it has been shown to inhibit tumor growth and promote apoptosis in a variety of hematologic tumors, gastric, cervical, breast, endometrial, and ovarian cancers [6–8]. Recent studies have confirmed that REA nanoparticles inhibit tumor cell migration, invasion by inhibiting matrix metalloproteinase-2 (MMP-2), 9 expressions, and angiogenesis in mouse breast cancer transplant tumors [9]. These studies demonstrated that REA is a potential antitumor agent with inhibitory effects on tumor cell proliferation, migration, and invasion. However, the effect of REA on EC intervention is not completely clear.

As research progressed, investigators identified a form of cell death characterized by iron-dependent accumulation of lipid reactive oxygen species-ferroptosis, and activation of ferroptosis inhibits tumor cell proliferation, while inhibition of glutathione peroxidase 4 (GPX4) activity selectively activates ferroptosis [10]. In addition, the ROS-ASK1-p38 MAPK signaling pathway is an important intracellular regulatory pathway of oxidative stress [11], and Hattori et al. [12] found that Erastin induced ferroptosis in a variety of mammalian cells by activating the ASK1-p38 axis downstream of lipid peroxidation accumulation. Ye et al. [13] found that HMGB1 induced massive production of lipid reactive oxygen species (ROS) and glutathione (GSH-PX) depletion, activating the RAS-JNK/p38 signaling pathway and inducing ferroptosis in cells. Thus, activation of the ROS-ASK1-p38 MAPK signaling pathway can lead to the ferroptosis of cells. However, it is not clear whether the ROS-ASK1-p38 MAPK signaling pathway is involved in the regulation of EC by REA, such as ferroptosis. Therefore, this study intends to provide a deeper understanding of the role of the ROS-ASK1-p38 MAPK pathway in the regulation of EC proliferation, migration, and ferroptosis by REA and to provide ROS-ASK1-p38 MAPK and ferroptosis based therapeutic targets for the treatment of EC.

## 2. Materials and Methods

### 2.1. Experimental Reagents

Human EC cell line Eca109 (no.CL-0077), KYSE150 (no.CL-0638) cells, and human normal esophageal epithelial cells HEEC (no. CP-H031) (Wuhan Procell Life Science and Technology Co., Ltd.), RPMI 1640 medium (no. G4530, Wuhan Servicebio Co., Ltd.), REA dry powder (no.SA4101, Hubei Norna Technology Co., Ltd.), CCK-8 kit (no.BS350 A, Biosharp, Shanghai), Crystalline Violet (no.C8470), ferroptosis inhibitor Ferrostatin-1 (Fer-1, no.IF0430), ferroptosis inducer Erastin (no.IE0310), apoptosis inhibitor Z-VAD- FMK (no. HY-16658B) (Beijing Solarbio Science & Technology Co., Ltd.), Matrigel (no.356234, Corning, USA), kits of malondialdehyde (MDA, no.ZC-S0343), superoxide dismutase (SOD, no.ZC-S0350), reduced glutathione (GSH, no.ZC-S0602), glutathione peroxidase (GPXS, no.ZC-S0860), ROS (no.ZC1126) (Shanghai ZCIBIO Technology Co., Ltd.), cell JC-1 assay kit (no. C2006, Shanghai Beyotime Biotechnology), TRIzol kits (no.15596018, Invitrogen, USA), Takara TB Green™ PreMix Ex Taq™ (no.RR820A, Takara), and experimental primary antibodies [E-cadherin (no.A3044), Slug (no.A1057), N-cadherin (no.A19083), ASK1 (no.A3271), p38 MAPK (no. A14401), p-p38 MAPK (no.A4771) and GPX4 (no.A11243)] were purchased from Wuhan ABclonal Technology Co., Ltd. Secondary antibody (horseradish peroxidation enzyme-labeled goat anti-rabbit antibody, no. ab6721) was purchased from Abcam, Inc., and BCA protein concentration determination kit (no. P0009, Beyotime Institute of Biotechnology), ECL luminescence kit (no.KF001, Affinity, USA), and Perls Prussian blue staining kit (no.M021, Shanghai Gefan Biotechnology Co., Ltd.) were prepared.

### 2.2. Experimental Instruments

DMI1 inverted biological microscope (LEICA, Germany), spectra max PLUS 384 enzyme marker (Molecular Devices, USA), CytoFLEX Flow analyzer (Beckman Coulter, Inc.), JY200C electrophoresis instrument (Beijing Junyi Electrophoresis Co., Ltd.), TE22 protein transmembrane instrument (Hoefer, USA), Panthera digital trinocular camera microscope (Motic China Group Co., Ltd.), and JEM-1400FLASH type transmission electron microscope (JEOL, Japan) were used.

### 2.3. Drug Preparation

The REA dry powder was dissolved in phosphate-buffered saline and stirred with a magnetic stirrer for 12 h. The suspension was filtered through a 0.2 *μ*m filter and stored at 4°C. Some of the samples were sent to the chemistry laboratory to determine the concentration of arsenic in the solution, and the concentration of arsenic in the solution was 5.498 mg/L as determined by ICP emission spectrometry.

### 2.4. Cell Culture

The cell lines Eca109 and KYSE150 were cultured in RPMI 1640 medium (containing 10% fetal bovine serum) with cell culture conditions of 5% CO_2_, 37°C, and the cells were digested with trypsin after growing to 70%–80% and then passaged. The experimental groupings were set as ① REA (0, 10, 20, 40, 60, 80, 100 *μ*mol/L), ② control, REA (1/2IC_50_, IC_50_, 2IC_50_), ③control, REA (2IC_50_), shRNA-ASK1, shRNA-NC, REA (2IC_50_) ^+^shRNA-ASK1, REA (2IC_50_) ^+^shRNA-NC, SB203580 (p38 MAPK inhibitor), REA (2IC_50_) ^+^SB203580 groups. HEEC cells were cultured in RPMI 1640 medium (containing 10% fetal bovine serum), culture conditions were as described above, and the experimental groupings were set up as follows: control, REA (1/2IC_50_, IC_50_, 2IC_50_).

### 2.5. shRNA Interference

The ASK1 shRNA and NC shRNA sequences were added along with Age I digestion sites and ligated with the pGC-FU vector after enzymatic digestion. The recombinant plasmids were then transfected into HEK293 T cells, positive cells were screened, and the plasmids were extracted. Eca109 and KYSE150 cells were inoculated onto 6-well plates, and cells were transfected after cell density reached 70%∼80% according to the instructions of lipofectamine 2000. The mixture was warmed at room temperature for 20 min and then added to the culture wells preinoculated with cells. Cells were incubated at 5% CO_2_, 37°C for 8 h to allow plasmid transfer into the cells, and then the cells were incubated in a complete medium for 24∼48 h for subsequent experiments.

### 2.6. CCK-8 Assay to Detect Cell Proliferation

Eca109 and KYSE150 cells at the logarithmic growth stage were taken, and the cell density was adjusted to 2 × 10^4^ cells/mL and inoculated in 96-well plates at 100 *μ*L per well. After adding different mass concentrations of REA for 24, 48, and 72 h, then 10 *μ*L CCK-8 solution was added to each well and mixed and incubated at 37°C for 2 h. The absorbance (A) values at 450 nm were measured using an enzyme marker, and the cell inhibition rate and half inhibition concentration (IC_50_) were calculated. Cell inhibition rate = [1-experimental group A/control group A] × 100%. HEEC cells in logarithmic growth phase were taken, REA was added at different mass concentrations, and cell proliferation was assayed as described above.

### 2.7. Clone Formation Assay to Detect Cell Proliferation Viability

Logarithmic growth phase Eca109 and KYSE150 cells were digested with trypsin and inoculated in 6-well plates at a cell density of 150 cells/well and incubated at 37°C in a 5% CO_2_ constant temperature incubator for 24 h. With 3 replicates in each group, add the corresponding concentrations of REA, and terminate the culture when the cell colonies were visible to the naked eye, use 4% paraformaldehyde to fix the cells for 30–60 min, 0.1% crystal violet staining for 5 min, discard the staining solution and rinse the cells with running water, let them dry naturally, take pictures and record, and count clones.

### 2.8. Scratch Assay to Detect Cell Migration Ability

Logarithmic growth stage Eca109 and KYSE150 cells were taken, and the cells were inoculated in 6-well plates with about 5 × 10^5^ cells per well, and on day 2, when cells grew to 100% fusion, a straight line of uniform strength and angle and thickness was lightly scratched on the bottom of the 6-well plate with a 10 *μ*L sterile gun tip (3 replicates per group). The width of the scratch in the same field was observed under an inverted phase contrast microscope at 0 and 24 h, respectively, and photographed.

### 2.9. Transwell Assay to Detect Cell Invasion

1 : 5 dilution of Matrigel, prechilled at 4°C, was added to the Transwell upper chamber, spread well, and dried at 37°C for 70 min. Groups were prepared cell suspensions, five replicate wells were set up for each group, and the cell concentration was adjusted to 5 × 105 cells/mL, 200 *μ*L of cell suspension was added to the upper chamber, and 500 *μ*L of medium containing 20% FBS was added to the lower chamber as a chemotactic factor. After adding REA, SB203580, or transfected shRNA-ASK1, the small chambers were incubated at 5% CO_2_ and 37°C for 24 h. The uninvaded cells in the upper chamber were wiped off with cotton swabs, rinsed with PBS, fixed with methanol, and stained with 0.1% crystal violet. 5 fields of view of each well were selected and photographed under a light microscope, and the number of migrated cells in each group was counted.

### 2.10. Western Blot Analysis

Eca109 and KYSE150 cells at the logarithmic growth stage were taken. Add the corresponding concentrations of REA, SB203580, or transfected shRNA-ASK1, and after 24 h of culture, cells were collected, and the total cellular protein was extracted using RIPA lysate, protein concentration was detected by BCA method, and protein was separated by 10% SDS-PAGE and transferred to PVDF membrane, which was closed with TBST containing 5% skim milk at room temperature for 2 h. Primary antibodies (E-cadherin, Slug, N-cadherin, ASK1, p38 MAPK, p-p38 MAPK, and GPX4, *β*-actin) were incubated overnight at 4°C, washed with TBST, and incubated with secondary antibodies at room temperature for 2 h and added to ECL luminescent solution for color development and photographed in an automatic exposure meter. The grayscale values of each protein band were analyzed by Image Pro Plus software, and the relative protein expression was calculated.

### 2.11. Quantitative Real-Time Polymerase Chain Reaction (qRT-PCR)

Eca109 and KYSE150 cells at the logarithmic growth stage were taken. Add the corresponding concentrations of REA, SB203580, or transfected shRNA-ASK1, and the cells were collected after 24 h of culture. Total RNA was extracted by lysing cells using the TRIzol kit according to the manufacturer's instructions and then reverse-transcribed to synthesize cDNA for qRT-PCR analysis. Gene expression levels were quantified using Takara TB Green ™PreMix Ex Taq™ with *β*-actin as an internal reference. qRT-PCR reaction conditions are as follows: initial denaturation at 95°C for 10 min, followed by denaturation at 95°C for 10 s, annealing at 60°C for 10 s, extension at 72°C for 10 s, 45 cycles, CT values were recorded using 2^−∆∆CT^ to analyze the relative expression levels. The primer sequences are shown in Table 1.

### 2.12. Detection of Mitochondrial Ultrastructure by Transmission Electron Microscopy

Logarithmic growth stage Eca109 and KYSE150 cells were taken. Add the corresponding concentrations of REA, SB203580, or transfected shRNA-ASK1, and the cells were collected after 24 h of culture, fixed with 2.5% glutaraldehyde for 12 h, 1% osmium acid for 2 h, embedded, sectioned, stained, and observed by transmission electron microscopy, and images were collected.

### 2.13. Prussian Blue Staining to Observe the Distribution of Intracellular Iron Particles

Eca109 and KYSE150 cells at the logarithmic growth stage were taken. Add the corresponding concentrations of REA, and the cells were collected after 24 h of incubation, fixed with 4% paraformaldehyde, incubated with Perl reagent, and stained, and then images were acquired by applying Panthera digital trinocular camera microscope.

### 2.14. Biochemical Kit Analysis

Eca109 and KYSE150 cells at the logarithmic growth stage were taken. Add the corresponding concentrations of REA, SB203580, or transfected shRNA-ASK1, and the cells were collected after 24 h of incubation. The supernatant was taken from the lysed cells, and the MDA content, SOD activity, GSH content, and GPXS activity were determined and calculated according to the kit instructions by biochemical method, and the optical density value of each concentration was detected by enzyme marker, and three parallel samples were set.

### 2.15. Flow Cytometric Analyses of ROS

Logarithmic growth stage Eca109 and KYSE150 cells were taken. Add the corresponding concentrations of REA, SB203580, or transfected shRNA-ASK1, and the cells were collected after 24 h of incubation, and then, 1 mL of DCFH-DA probe working solution at a final concentration of 10 *μ*mol/L was added and incubated for 20 min at 37°C. The fluorescence intensity was quantified by flow cytometry to reflect the ROS content in each cell group (excitation wavelength 488 nm, emission wavelength 525 nm).

### 2.16. Immunofluorescence Assay

Cells grown to log phase were inoculated at 4.5 × 10^4^ into 6-well plates overnight and treated with REA, SB203580, or transfected shRNA-ASK1 for 24 h. Cells were washed, and 4% paraformaldehyde fixed cells, 0.25% Triton × 100 permeable membrane, 10% goat serum closed, and primary antibody (GPX4) were added overnight at 4°C and washed, and the secondary antibody was added and incubated at room temperature for 2 h, washed, and photographed by inverted fluorescence microscopy.

### 2.17. Detection of Mitochondrial Membrane Potential by the JC-1 Method

Logarithmic growth stage Eca109 and KYSE150 cells were taken and treated with REA, SB203580, or transfected shRNA-ASK1 for 24 h according to the grouping, and each well was incubated for 20 min at 37°C with 1 mL of JC-1 staining solution and 1 mL of culture solution. The cells were washed twice with JC-1 staining buffer after incubation, the cells were collected by trypsin digestion, and the cell fluorescence intensity was detected by flow cytometry to calculate the proportion of depolarized cells.

### 2.18. Statistical Analysis

Data were statistically analyzed using SPSS 22.0 statistical software (IBM Corp), and dates were expressed as mean ± standard error of the mean (SEM), and LSD-*t* test was used to analyze the data with only two groups, and one-way ANOVA of variance was used to analyze the differences among multiple groups, with *P* < 0.05 indicating that the differences were statistically significant.

## 3. Results

### 3.1. Effect of REA on the Proliferation of EC Cells

To observe the effect of REA on the proliferation of EC cells, we examined the effect of different concentrations of REA on the proliferation of Eca109 and KYSE150 cells. The results showed that the proliferation of Eca109 and KYSE150 cells slowed down as the concentration of REA increased, the inhibition rate of Eca109 and KYSE150 cells increased with time under the same conditions of REA concentration, and the IC_50_ of REA effect on Eca109 and KYSE150 cells were 61.336 *μ*mol/L and 48.012 *μ*mol/L, respectively. In addition, no significant changes in cell proliferation were observed when REA with IC_50_ of 61.336 *μ*mol/L and 48.012 *μ*mol/L was applied to HEEC cells, respectively (Figure 1). These results indicated that REA markedly inhibited the proliferation of EC cells and was not toxic to HEEA cells.

### 3.2. Effect of REA on the Migration and Invasion of EC Cells

To determine the extent of cell migration and invasion after REA treatment, the cells were observed by scratch and Transwell assays. Compared with the control group, the REA 1/2IC_50_, IC_50_, and 2IC_50_ groups significantly slowed down the planar migration ability of Eca109 and KYSE150 cells, and at 24 h, the control group Eca109 and KYSE150 cells were almost completely fused, while the migration of Eca109 and KYSE150 cells in the REA 1/2IC_50_, IC_50_ and 2IC_50_ groups was significantly reduced (*P* < 0.05, Figures 2(a) and 2(b)). The number of cell invasions was distinctly reduced in the Eca109 and KYSE150 cells in the REA 1/2IC_50_, IC_50_, and 2IC_50_ groups (*P* < 0.01, Figures 2(c) and 2(d)). The protein expression of Slug and N-cadherin was markedly decreased in the Eca109 and KYSE150 cells in the REA IC_50_ and 2IC_50_ groups, while the protein expression of E-cadherin was distinctly increased in the Eca109 and KYSE150 cells in the REA IC_50_ and 2IC_50_ groups (*P* < 0.05, Figure 2(e)). These data indicated that REA markedly inhibited cell migration and invasion of EC cells.

### 3.3. Effect of REA on Ferroptosis in EC Cells

The ferroptosis indexes in cells were analyzed to evaluate the effect of REA on ferroptosis in EC cells. Compared with the control group, a large number of mitochondria in the cytoplasm of Eca109 and KYSE150 cells in the REA 2IC_50_ group underwent swelling and autophagy, the rough endoplasmic reticulum expanded, and the mitochondrial cristae became shorter and fewer or even disappeared (Figure 3(a)). The results of Prussian blue staining showed that there were no blue-stained granules in the control group, and blue-stained granules of different sizes and amounts could be found in Eca109 and KYSE150 cells in the REA 1/2IC_50_, IC_50_, and 2IC_50_ groups (Figure 3(b)). Compared with the control group, the fluorescence intensity of ROS and SOD, GSH, and GPXS activity were significantly increased in Eca109 and KYSE150 cells in the REA 1/2IC_50_, IC_50_, and 2IC_50_ groups, whereas MDA activity and expression of GPX4 were markedly decreased in Eca109 and KYSE150 cells in the REA IC_50_ and 2IC_50_ groups (*P* < 0.05, Figures 3(c)–3(g)). These results indicated that REA induced ferroptosis in EC cells.

### 3.4. Effect of REA on ROS/ASK1/p38 MAPK Signaling Pathway in EC Cells

In order to determine the changes of ROS/ASK1/p38 MAPK signal pathway EC cells after REA intervention, we detected the expression levels of ASK1, p38 MAPK, and p-p38 MAPK. Compared with the control group, the mRNA expression of ASK1 and p38 MAPK was significantly increased in Eca109 and KYSE150 cells in the REA IC_50_ and 2IC_50_ groups (Figure 4(a)), whereas the protein expression of ASK1 and p-p38 MAPK was markedly increased in Eca109 and KYSE150 cells in the REA IC_50_ and 2IC_50_ groups (*P* < 0.05), and the protein expression of p38 MAPK was not significant in KYSE150 cells in the REA 1/2IC_50_, IC_50_ and 2IC_50_ groups (*P* > 0.05, Figures 4(b) and 4(c)). These results demonstrated that REA increased the mRNA and protein levels of related factors in the ROS/ASK1/p38 MAPK pathways.

### 3.5. Effect of Ferroptosis Activation on Migration and Invasion of EC Cells

Next, we analyzed the effect of ferroptosis activation on the migration and invasion of EC cells. A large number of mitochondria in the cytoplasm of Eca109 and KYSE150 cells in the REA 2IC_50_ and 2IC_50_^+^Erastin groups became swollen and autophagic, and the rough endoplasmic reticulum expanded, and the mitochondrial cristae became shorter and fewer or even disappeared (Figure 5(a)). Compared with the control group, the migration and invasion of Eca109 and KYSE150 cells in the 2IC_50_, 2IC_50_^+^Fer-1, 2IC_50_^+^ZVAD-FMK, and 2IC_50_^+^Erastin groups were distinctly reduced (*P* < 0.01); compared with the 2IC_50_ group, the migration and invasion of Eca109 and KYSE150 cells in the 2IC_50_^+^Fer-1, 2IC_50_^+^ZVAD-FMK groups were significantly increased, and in the 2IC_50_^+^Erastin group, they were significantly decreased (*P* < 0.05, Figures 5(b)–5(e)). Compared with the control group, the protein expression of Slug and N-cadherin was markedly decreased in the Eca109 and KYSE150 cells in the 2IC_50_ and 2IC_50_^+^Erastin groups, while the protein expression of E-cadherin was distinctly increased in the Eca109 and KYSE150 cells in the 2IC_50_, 2IC_50_+Fer-1, and 2IC_50_+Erastin groups (*P* < 0.05); compared with the 2IC_50_ group, the protein expression of Slug and N-cadherin was markedly decreased in the Eca109 and KYSE150 cells in the 2IC_50_^+^Erastin group, while the protein expression of E-cadherin was distinctly increased in the Eca109 and KYSE150 cells in the 2IC_50_+Erastin group (*P* < 0.05, Figure 5(f)). These results indicated that ferroptosis activation promotes the inhibitory effect of REA on EC cell migration and invasion.

### 3.6. Effect of Inhibiting ROS/ASK1/p38 MAPK Signaling Pathway on Migration and Invasion in REA-Treated EC Cells

The function of the ROS/ASK1/p38 MAPK signaling pathway in REA inhibition of EC cell migration was validated using shRNA interference vectors (shRNA-ASK1) and inhibitors (SB203580). Compared with the control group, the migration and invasion of Eca109 and KYSE150 cells in the 2IC_50_, shRNA-ASK1, 2IC_50_+shRNA-ASK1, 2IC_50_+shRNA-NC, SB203580, and 2IC_50_+ SB203580 groups were distinctly reduced (*P* < 0.01), and the protein expression of ASK1, p38 MAPK, p-p38 MAPK, Slug, and N-cadherin was markedly decreased in Eca109 and KYSE150 cells in the shRNA-ASK1, 2IC_50_^+^shRNA-ASK1, SB203580, and 2IC_50_^+^SB203580 groups, whereas the protein expression of E-cadherin was significantly increased in Eca109 and KYSE150 cells in the shRNA-ASK1, 2IC_50_^+^shRNA-ASK1, SB203580, and 2IC_50_^+^SB203580 groups (*P* < 0.05). Compared with the 2IC_50_ group, the migration and invasion and the protein expression of ASK1, p38 MAPK, p-p38 MAPK, Slug, and N-cadherin of Eca109 and KYSE150 cells in the 2IC_50_^+^shRNA- ASK1 and 2IC_50_^+^SB203580 groups were observably decreased, and the protein expression of E-cadherin was markedly increased in Eca109 and KYSE150 cells in the 2IC_50_^+^shRNA-ASK1 and 2IC_50_+SB203580 groups (*P* < 0.05). Compared with the shRNA-ASK1 group, the migration and the protein expression of Slug and N-cadherin of Eca109 and KYSE150 cells in the 2IC_50_^+^shRNA- ASK1 and 2IC_50_+SB203580 groups were prominently decreased, and the protein expression of ASK1, p38 MAPK, p-p38 MAPK, and E-cadherin was notably increased in Eca109 and KYSE150 cells in the 2IC_50_+shRNA-ASK1 and 2IC_50_+SB203580 groups (*P* < 0.05) (Figures 6(a)–6(g)). These results demonstrated that the inhibition of the ROS/ASK1/p38 MAPK signaling pathway promotes REA inhibition of EC cell migration and invasion.

### 3.7. Effect of Inhibition of ROS/ASK1/p38 MAPK Signaling Pathway on Ferroptosis in REA-Treated EC Cells

Further, we determined the effect of inhibition of ROS/ASK1/p38 MAPK signaling pathway on ferroptosis in REA-treated EC cells. Eca109 and KYSE150 cells in the 2IC_50_, 2IC_50_^+^shRNA-ASK1, and 2IC_50_^+^SB203580 group's mitochondria were swollen and autophagic, the rough endoplasmic reticulum was dilated, and mitochondrial cristae were shortened and reduced or even disappeared (Figure 7(a)). Compared with the control group, the fluorescence intensity of ROS and SOD, GSH, and GPXS activity were significantly increased in Eca109 and KYSE150 cells in the 2IC_50_, shRNA-ASK1, 2IC_50_^+^shRNA-ASK1, 2IC_50_^+^shRNA-NC, SB203580, and 2IC_50_^+^SB203580 groups, whereas JC-1 red/green percentage, MDA activity, and mRNA and protein expression of GPX4 were markedly decreased in Eca109 and KYSE150 cells in the 2IC_50_, shRNA-ASK1, 2IC_50_^+^shRNA-ASK1, 2IC_50_^+^shRNA-NC, SB203580, and 2IC_50_^+^SB203580 groups (*P* < 0.05). Compared with the shRNA- ASK1 group, the fluorescence intensity of ROS was observably increased in Eca109 and KYSE150 cells in the 2IC_50_^+^shRNA-ASK1 and 2IC_50_^+^SB203580 groups, whereas JC-1 red/green percentages were dramatically decreased in KYSE150 cells, and the mRNA expression of GPX4 was markedly reduced in Eca109 cells in the 2IC_50_+shRNA-ASK1 and 2IC_50_+SB203580 groups (*P* < 0.05). Compared with the SB203580 group, the fluorescence intensity of ROS was significantly increased, and JC-1 red/green percentages were markedly decreased in Eca109 and KYSE150 cells in the 2IC_50_+SB203580 group (*P* < 0.05) (Figures 7(b)–7(h)). These results suggested that the inhibition of the ROS/ASK1/*p*38 MAPK signaling pathway promotes ferroptosis in REA-treated EC cells.

## 4. Discussion

In the present study, we demonstrated that REA was not significantly toxic to HEEC cells, inhibited proliferation, migration, and invasion of Eca109 and KYSE150 cells, and also induced ferroptosis and activated the ROS/ASK1/p38 MAPK signaling pathway in Eca109 and KYSE150 cells. Further results showed that induction of ferroptosis promoted the inhibitory effects of REA on EC cell migration and invasion, and inhibition of the ROS/ASK1/p38 MAPK signaling pathway promoted REA inhibition of EC cell migration, invasion, and induction of ferroptosis. Thus, it is evident that the inhibition of cell migration, invasion, and induction of ferroptosis by REA may be achieved by inhibiting the ROS/ASK1/p38 MAPK signaling pathway.

To date, EC is still a challenge to treat [14]. It has previously been observed that REA significantly inhibited breast cancer cell migration and invasion *in vitro* and lung and liver metastasis *in vivo* [9]. In addition, REA inhibits migration and invasion of gastric cancer cells by blocking tumor cell adhesion and reducing the ability of tumor cells to destroy the basement membrane [15]. In our study, we found that the proliferation of Eca109 and KYSE150 cells showed a decreasing trend depending on the increasing concentration of REA, and the IC_50_ of its effect on Eca109 and KYSE150 cells was 61.336 *μ*mol/L and 48.012 *μ*mol/L, respectively. Therefore, 1/2IC_50_, IC_50_, and 2IC_50_ were used as the REA treatment in this study concentration. Extensive research has shown that epithelial mesenchymal transition (EMT) is a key process in tumor metastasis, E-cadherin inhibits EMT, Slug promotes EMT-induced cell migration, and N-cadherin is highly expressed in esophageal squamous carcinoma tissues, which is also associated with tumor metastasis [16]. In this experiment, we found that REA was not significantly toxic to HEEC cells, and REA IC_50_ and 2IC_50_ could significantly increase the expression of E-cadherin and reduce the expression of Slug and N-cadherin in EC cells, and scratch assay and Transwell assay also showed that REA significantly decreased cell migration and cell invasion. These findings confirmed that REA has the effect of inhibiting the proliferation, migration, and invasion of EC cells.

There is a growing body of literature that recognizes activation of ferroptosis can inhibit tumor cell proliferation [17], and GPX4, a phospholipid hydroperoxide glutathione peroxidase, can inhibit ferroptosis in tumor cells [18]. Prior studies have noted that GPX4 is highly expressed in hepatocellular carcinoma and colon cancer and that high GPX4 expression is a poor prognostic factor in diffuse large B-cell lymphoma and lung adenocarcinoma [19,20]. Zhang et al. [21] showed that GPX4 activity was reduced in esophageal cancer TE1 cells after oridonin administration and was consistent with intracellular Fe^2+^, lipid peroxidation products, MDA, and ROS accumulation after oridonin. A similar mechanism was reported by Shishido et al. [22] who demonstrated that GPX4 upregulation is a poor prognostic factor in esophageal squamous cell carcinoma. In the present study, REA IC_50_ and 2IC_50_ caused significant downregulation of GPX4 and decreased MDA content and increased SOD, GSH, and GPXS activities in EC cells, and cellular mitochondria underwent swelling, autophagy, and the discovery of blue-stained granules of various sizes and amounts. This indicates that REA may induce ferroptosis in Eca109 and KYSE150 cells. To further investigate whether ferroptosis affects the inhibitory effect of REA on migration and invasion of Eca109 and KYSE150, we first treated EC cells with REA and then treated the cells with ferroptosis inhibitor (Fer-1), ferroptosis inducer (Erastin), and apoptosis inhibitor (Z-VAD-FMK). The present results showed that the migration and invasion of Eca109 and KYSE150 cells were significantly inhibited in the 2IC_50_^+^Erastin group, while the migration and invasion of cells were significantly increased in the 2IC_50_^+^Fer-1 and 2IC_50_^+^ZVAD-FMK groups, and 2IC_50_^+^ Erastin significantly decreased the protein expression of Slug and N-cadherin and significantly increased the protein expression of E-cadherin in Eca109 and KYSE150 cells; taken altogether, these results indicate that ferroptosis activation promotes the inhibitory effect of REA on EC cell migration and invasion.

Oxidative stress can mediate the activation of multiple intracellular pathways, such as MAPK and NF-*κ*B, which have crossover and feedback and influence each other [23]. MAPK is a class of serine/threonine protein kinases that can transmit exogenous signals down through a multistage protein kinase cascade reaction, which in turn regulates genetic and cellular physiological responses in response to environmental changes, and is an important cellular signal transduction pathway that responds to oxidative stress [24]. Four MAPK family members have been identified, that is, p38 MAPK, JNK, ERK1/2, and ERK5, which can play important roles in the regulation of cell growth, differentiation, and apoptosis [25]. The p38 MAPK is stimulated and activated by cytokines and environmental stress and belongs to stress-activated protein kinases, which are involved in regulating cell proliferation, differentiation, and apoptosis [26]. ASK1, a member of the MAP3K family, is ROS-sensitive and is a key gene in oxidative stress-mediated apoptosis [27]. After oxidative stress, the Thr 845 site of ASK1 is phosphorylated and then activated, and activated ASK1 can phosphorylate downstream MKK4 and MKK7, which can phosphorylate downstream MKK3 and MKK6, which activate p38 by phosphorylating Thr180 and Tyr182 [28, 29]. Therefore, the ROS-ASK1-p38 MAPK signaling pathway is an important intracellular regulatory pathway for oxidative stress. Ye et al. [13] found that HMGB1 induced massive production of lipid reactive oxygen species (ROS) and glutathione (GSH-PX) depletion, activating the RAS-JNK/p38 signaling pathway and inducing ferroptosis in cells. Wang et al. [30] found that REA induced apoptosis and autophagy in osteosarcoma cells through activation of ROS/JNK and inhibition of the Akt/mTOR signaling pathway. In this experiment, we confirmed that the expression of ASK1, p38 MAPK, and p-p38 MAPK increased significantly in REA IC_50_ and 2IC_50_ of Eca109 and KYSE150 cells. Moreover, the migration, invasion, the mRNA expression of GPX4, and the protein expression of Slug and N-cadherin were observably decreased, and the fluorescence intensity of ROS and the protein expression of E-cadherin were markedly increased of Eca109 and KYSE150 cells in the 2IC_50_^+^shRNA-ASK1 and 2IC_50_^+^SB203580 groups. This may indicate that REA induces ferroptosis and inhibits cell migration in EC cells by activating the ROS-ASK1-p38 MAPK signaling pathway.

In conclusion, these observations suggest that REA dose-dependently inhibited the proliferation of Eca109 and KYSE150 cells, suppressed cell migration and invasion, induced cellular ferroptosis, and activated the ROS-ASK1-p38 MAPK signaling pathway. After treatment with REA + shRNA-ASK1 or SB203580, the signal of ROS-ASK1-p38 MAPK and the cell migration and invasion were inhibited, and cellular ferroptosis was promoted. This study provides a basis for the study of the Chinese herbal medicine REA, a method for the treatment of EC, and an experimental foundation for the exploration of new targets for the treatment of EC.

## Figures and Tables

**Figure 1:** Effect of REA on the proliferation of EC cells. (a) Cell inhibition rates of Eca109 and KYSE150 cells were treated with REA with the concentration of 0, 10, 20, 40, 60, 80, and 100 *μ*mol/L for 24 h, 48 h, and  72h; (b, c) clone formation assay was performed to detect the proliferation viability of Eca109 and KYSE150 cells treated with REA at concentrations of 0, 10, 20, 40, 60, 80, and 100 *μ*mol/L; (d) detection of proliferation viability of HEEC cells treated with REA at IC_50_ concentrations of 61.336 *μ*mol/L and 48.012 *μ*mol/L. The data are expressed as the mean ± SD. Compared with the 0 *μ*mol/L, ^*∗∗*^*P* < 0.05.

**Figure 2:** Effect of REA on the migration and invasion of EC cells. (a) Results of Eca109 and KYSE150 cells scratch assay (scale bar, 100 *μ*m); (b) Eca109 and KYSE150 cells migration; (c) Transwell invasion assay of Eca109 and KYSE150 cells (crystal violet staining, 400x, Scale bar, 50 *μ*m); (d) number of membrane piercing in Eca109 and KYSE150 cells; (e) the expression of E-cadherin, Slug, and N-cadherin in Eca109 and KYSE150 cells was determined using western blot analysis. The data were expressed after being normalized to *β*-actin. The data are expressed as the mean ± SD. Compared with the control group, ^*∗*^*P* < 0.05 and ^*∗∗*^*P* < 0.01.

**Figure 3:** Effect of REA on ferroptosis in EC cells. (a) Transmission electron microscopy observation of Eca109 and KYSE150 cells (15000x, scale bar, 500 nm); (b) Eca109 and KYSE150 cells-Prussian blue staining (400x, scale bar, 50 *μ*m and 200 *μ*m); (c) flow cytometric analysis of Eca109 and KYSE150 cells ROS; (d) ROS fluorescence intensity of Eca109 and KYSE150 cells; (e) Eca109 and KYSE150 cells GPX4 immunofluorescence staining (40x, Scale bar, 20 *μ*m); (f) GPX4 expression in Eca109 and KYSE150 cells; (g) the content of MDA, SOD, GSH, and GPXS in Eca109 and KYSE150 cells. The data are expressed as the mean ± SD. Compared with the control group, ^*∗*^*P* < 0.05 and ^*∗∗*^*P* < 0.01.

**Figure 4:** Effect of REA on ROS/ASK1/p38 MAPK signaling pathway in EC cells. (a) Relative mRNA expression of ASK1 and p38 MAPK; (b) relative protein expression of ASK1, p38 MAPK, and p-p38 MAPK; (c) protein band calculated as a ratio relative to *β*-actin protein levels. The data are expressed as the mean ± SD. Compared with the control group, ^*∗*^*P* < 0.05 and ^*∗∗*^*P* < 0.01.

**Figure 5:** Effect of ferroptosis activation on migration and invasion of EC cells. (a) Transmission electron microscopy observation of Eca109 and KYSE150 cells (15000x, scale bar, 500 nm); (b) results of Eca109 and KYSE150 cells scratch assay (Scale bar, 100 *μ*m); (c) Transwell invasion assay of Eca109 and KYSE150 cells (crystal violet staining, 400x, Scale bar, 50 *μ*m); (d) Eca109 and KYSE150 cells migration; (e) the number of membrane piercing in Eca109 and KYSE150 cells; (f) the expression of E-cadherin, Slug, and N-cadherin in Eca109 and KYSE150 cells was determined using western blot analysis. The data were expressed after being normalized to *β*-actin. The data are expressed as the mean ± SD. Compared with the control group, ^*∗*^*P* < 0.05 and ^*∗∗*^*P* < 0.01; compared with the 2IC50 group, ^#^*P* < 0.05 and ^##^*P* < 0.01.

**Figure 6:** Effect of inhibiting ROS/ASK1/p38 MAPK signaling pathway on migration and invasion in REA-treated EC cells. (a) Eca109 and KYSE150 cells migration; (b) number of membrane piercing in Eca109 and KYSE150 cells; (c) results of Eca109 and KYSE150 cells scratch assay (scale bar, 100 *μ*m); (d) Transwell invasion assay of Eca109 and KYSE150 cells (crystal violet staining, 400x, Scale bar, 50 *μ*m); (e) protein band calculated as a ratio relative to *β*-actin protein levels; (f) relative protein expression of ASK1, p38 MAPK, and p-p38 MAPK; (g) relative protein expression of E-cadherin, Slug, and N-cadherin. The data are expressed as the mean ± SD. Compared with the control group, ^*∗*^*P* < 0.05 and ^*∗∗*^*P* < 0.01; compared with the 2IC50 group, ^#^*P* < 0.05 and ^##^*P* < 0.01; compared with the shRNA-ASK1 group, ^Δ^*P* < 0.05 and ^ΔΔ^*P* < 0.01; compared with the SB203580 group, ^▲^P<0.05 and ^▲▲^*P* < 0.01.

**Figure 7:** Effect of inhibition of ROS/ASK1/*p*38 MAPK signaling pathway on ferroptosis in REA-treated EC cells. (a) Transmission electron microscopy observation of Eca109 and KYSE150 cells (15000x, scale bar, 500 nm); (b) flow cytometric analysis of Eca109 and KYSE150 cells ROS; (c) results of flow cytometric detection of changes in the mitochondrial membrane potential of Eca109 and KYSE150 cells; (d) ROS fluorescence intensity of Eca109 and KYSE150 cells; (e) JC-1 red/green percentage of Eca109 and KYSE150 cells; (f) the content of MDA, SOD, GSH, and GPXS in Eca109 and KYSE150 cells; (g) the mRNA expression of GPX4 in Eca109 and KYSE150 cells; (h) the protein expression of GPX4 in Eca109 and KYSE150 cells. The data were expressed after being normalized to *β*-actin. The data are expressed as the mean ± SD. Compared with the control group, ^*∗*^*P* < 0.05 and ^*∗∗*^*P* < 0.01; compared with the 2IC50 group, ^#^*P* < 0.05 and ^##^*P* < 0.01; compared with the shRNA-ASK1 group, ^Δ^*P* < 0.05 and ^ΔΔ^*P* < 0.01; compared with the SB203580 group, ^▲^*P* < 0.05 and ^▲▲^*P* < 0.01.

**Table 1:** Primer sequences.

Primer	Forward primer (5′-3′)	Reverse primer (5′-3′)
*ASK1*	CGTAGCCTCTTGGTCCTTTATC	GGAAGTCTTTCTGCTCTCCTTC
*p38 MAPK*	GCCTCACCGCCTCAGTAT	GCAGTCTTCTCATTCCCTTG
*GPX4*	ATACGCTGAGTGTGGTTTGC	CTTCATCCACTTCCACAGCG
*β*-Actin	CTCCATCGTCCACCGCAAATGCTTCT	GCTCCAACCGACTGCTGTCACCTTC

## Data Availability

The datasets used or analyzed during the current study are available from the corresponding author upon reasonable request.
